This article has been retracted.

# Effects and Clinical Value of Peritoneal Dialysis on Water and Water Balance, Adverse Reactions, Quality of Life, and Clinical Prognosis in Patients with Decompensated Chronic Nephropathy: A Systematic Review and Meta-Analysis

**DOI:** 10.1155/2022/9469134

**Published:** 2022-07-18

**Authors:** Xichao Wang, Miaomiao Zhang, Na Sun, Wenxiu Chang

**Affiliations:** Department of Nephrology, Tianjin First Central Hospital, Tianjin 300192, China

## Abstract

**Objective:**

To systematically evaluate the effects of peritoneal dialysis and hemodialysis on renal function and quality of life in patients with end-stage renal disease. An evidence-based medical rationale would be provided for peritoneal dialysis or hemodialysis treatment in patients with end-stage renal disease.

**Methods:**

The PubMed, EMBASE, ScienceDirect, Cochrane Library, China National Knowledge Infrastructure (CNKI), China VIP Database, Wanfang, and China Biomedical Literature Database (CBM) online databases were searched. Comparisons on the effects of peritoneal dialysis on renal function and quality of life were taken between patients with end-stage renal disease (RD). The data were extracted independently by two researchers. The bias-risk-included literatures were assessed according to the Cochrane manual 5.1.0 standard. RevMan 5.4 statistical software was used to analyze the collected data via meta-analysis.

**Results:**

Seven RCT articles were finally included. A total of 745 samples were analyzed via meta-analysis. The obvious heterogeneities of serum creatinine (Scr) and blood urea nitrogen (BUN) were discovered (*P* < 0.00001) in the selective investigations. According to the results of this analysis, it was indicated that the renal function of patients with end-stage renal disease treated by peritoneal dialysis was significantly better than that of hemodialysis. According to the meta-analysis, there was obvious heterogeneity of life quality among the included research data. It was indicated that the score of quality of life of patients with end-stage renal disease treated by peritoneal dialysis was significantly better than that of hemodialysis.

**Conclusion:**

Compared with hemodialysis in the treatment of end-stage renal disease, the renal function and quality of life of patients with peritoneal dialysis are better than those of hemodialysis. More further studies and follow-up with higher methodological quality and longer intervention time are still needed for further verification.

## 1. Introduction

End-stage renal disease (ESRD) has become a global public problem threatening human health. Recently, the Global Kidney Health Map (Global Kidney Health Atlas) published by the International Society of Nephrology (ISN) has displayed that there will be 14.5 million end-stage renal disease (ESKD) patients in the world by 2030. However, 5.4 million ESKD patients will be unable to receive treatment due to various factors. In low-income countries, ESKD patients are less likely to receive dialysis or kidney transplantation than in high-income countries. At present, with the development of blood purification technology and the popularization of medical insurance policy, the proportion of ESRD patients choosing dialysis treatment is also gradually increasing [1]. A British study found that the number of dialysis patients aged ≥65 increased by 29%, which was higher than the 16% growth rate of young and middle-aged dialysis patients aged 18 to 65 from 2005 to 2008 [2]. The age of patients who underwent their first dialysis is mainly over 65 years old, among which the number of patients over 75 years old increases rapidly and the proportion of elderly patients over 80 years old increases by 57% [3]. In South Korea, the average age of dialysis patients increased from 55.2 in 2005 to 58 in 2010 [4]. Hemodialysis (HD) and peritoneal dialysis (PD) are the most important methods of renal replacement therapy [5]. In recent years, some studies have compared the survival rates of the two dialysis methods, but the conclusions are controversial. It has been reported that in the early stage of dialysis, the survival rate of PD patients is better than that of HD patients [6]. Other studies show that the survival rates of the two groups of dialysis patients are similar [7].

As we all know, the main ways of clinical treatment of end-stage renal disease include renal replacement therapy and nondialysis therapy, in which renal replacement therapy includes hemodialysis, peritoneal dialysis, and renal transplantation [8]. For ESRD patients, due to their own basic diseases, poor economic strength, kidney tension, and other factors, most patients cannot receive transplantation treatment. Therefore, most clinical ESRD patients rely on dialysis to maintain their lives, mainly hemodialysis. The data show that up to 89.5% of patients in China regularly receive maintenance hemodialysis (MHD) as renal replacement therapy [9–11]. Hemodialysis is the main renal replacement therapy for patients with acute and chronic renal failure, which can effectively expel metabolic waste from the body and maintain the stability of the internal environment. Although hemodialysis technology is becoming more and more perfect, some uremic symptoms can be alleviated by dialysis [12]. MHD patients often have different degrees of malnutrition due to anorexia, digestive dysfunction caused by toxin accumulation, and nutrient loss caused by dialysis itself. Moreira et al. reported that the incidence of malnutrition in dialysis patients was as high as 93.8%, of which 81.5% were mild malnutrition and 12.3% were moderately malnourished [13]. Malnutrition is related to fatigue, cognitive impairment, and decreased physical activity, which affects the prognosis of patients. Peritoneal dialysis was first translated into Chinese in 1960 and did not enter the Chinese market until the late 1990s [14, 15]. In many countries, the prognosis of PD patients is equal to or better than that of HD [16, 17]. Based on this, this study focused on the effect of peritoneal dialysis compared with hemodialysis on renal function and quality of life in patients with end-stage renal disease to provide evidence-based medicine for patients with end-stage renal disease to choose peritoneal dialysis or hemodialysis treatment.

## 2. Research Contents and Methods

### 2.1. Sources and Retrieval Methods of Documents

China National Knowledge Infrastructure Network, China Biomedical Literature Database, VIP Database, Wanfang Database, Cochrane Library, PubMed, EMBASE, and Web of Science were searched. The search time limit was the beginning for each database until Feb. 28, 2022. This study applied the strategy of combining subject words, key words, and free words for literature retrieval. English key words consisted of end-stage renal disease, chronic renal failure, chronic uremia, peritoneal dialysis, hemodialysis, quality of life, and renal function.

### 2.2. Inclusion and Exclusion Criteria of Literature

#### 2.2.1. Literature Inclusion Criteria

1. Study types were cross-sectional studies, case-control studies, and cohort studies, regardless of blind or distributive concealment
2. Case inclusion criterion were as follows: (1) age ≥ 18 years old; (2) accord with end-stage renal disease diagnosis, eGFR < 15 ml/(min · 1.73 m^2^); (3) renal replacement therapy for more than 3 months: HD or PD; and (4) fluent writing and language communication
3. Case exclusion criterion were as follows: (1) clinically clear history of cerebrovascular disease or mental illness, (2) visual or hearing impairment or other sensory or motor disorders, (3) history of alcohol poisoning, and (4) recent acute disease or hospitalization
4. Intervention measures included hemodialysis and peritoneal dialysis. The renal function and quality-of-life scores of patients with different renal replacement therapies were compared

#### 2.2.2. Literature Exclusion Criteria

(1) It was not a randomized controlled study. (2) The data report was incomplete, and the data could not be used. (3) The research content and the latest research were repeated. (4) The evaluation of the efficacy of the study was not limited to the scores of renal function and quality of life in patients with end-stage renal disease.

### 2.3. Quality Evaluation and Data Extraction

Data extraction was obtained by the screening of two researchers in strict accordance to the inclusion and exclusion criteria. In addition, the extracted data was checked by a third party. The extracted contents included (1) the author's name and publication time; (2) the basic data, sample size and, dialysis time of the two groups; and (3) the changes of curative effect index data and adverse events pre- and posttreatment.

The literature quality evaluation was as follows: the literature quality was evaluated according to the Cochrane Collaboration Network risk-of-bias assessment tool recommended by the Cochrane Handbook version 5. 1. 0.

### 2.4. Statistical Processing

RevMan 5.3 software was used for meta-analysis. Because the meta-analysis outcome evaluation index (quality of life, renal function) was a continuous variable, the outcome index evaluation scale of each study was different. So the standardized mean difference (SMD) was used as the effect index and the point estimate and 95% CI were given for each effect. The chi-square test was used to determine whether there was heterogeneity between studies. When *P* ≥ 0.1 and *I*^2^ < 50%, no heterogeneity could be considered and the fixed-effect model should be selected. When *P* < 0.1 and *I*^2^ ≥ 50%, the sensitivity analysis should be used to find out the source of heterogeneity as much as possible. If heterogeneity could not be eliminated, the random-effect model should be used. The studies with obvious clinical heterogeneity were analyzed by subgroup analysis or sensitivity analysis or only by descriptive analysis.

## 3. Results and Analysis

### 3.1. The Results of Literature Retrieval and the Basic Situation of Literature Inclusion

2422 articles were retrieved through the computer databases. 324 articles were obtained after eliminating repeated studies. 133 articles were obtained from preliminary reading of titles and abstracts. 32 articles were included after excluding irrelevant studies, reviews, case reports, and noncontrol literatures. Then, 25 articles with incomplete data and no main outcome indicators were read carefully. Finally, 7 RCTs were included [18–24]. A total of 745 samples were analyzed via meta-analysis. The basic features included in the literature are shown in Table 1.

### 3.2. Evaluation of the Quality of the Methodology Included in the Literature

All the 7 RCT literatures included in this meta-analysis reported the baseline of patients. Only 3 RCTs mentioned “random assignment” without any explanation, and the rest did not mention “random” information. The seven studies included all gave detailed intervention measures and follow-up time. The number and reasons of the blind method and lost follow-up or withdrawal were not described in detail in 7 RCT articles. The risk-of-bias analysis is shown in Figures 1 and 2.

### 3.3. Results of Meta-Analysis

#### 3.3.1. Renal Function

Through a total of 745 samples on 7 RCTs, the renal function between the experimental group and the control group was analyzed via meta-analysis. Obvious heterogeneity of serum creatinine (Scr) was found among the included research data (chi^2^ = 44.95, df = 4, *P* < 0.00001, *I*^2^ = 91%). Obvious heterogeneity of blood urea nitrogen (BUN) was found among the included research data (chi^2^ = 32.32, df = 3, *P* < 0.00001, *I*^2^ = 91%). According to the results of this analysis, it is considered that there is a statistical difference in renal function between peritoneal dialysis and hemodialysis in patients with end-stage renal disease, indicating that the renal function of patients with end-stage renal disease treated by peritoneal dialysis is significantly better than that of hemodialysis. All the results are shown in Figures 3 and 4.

#### 3.3.2. Quality-of-Life Score

Through the 7 included RCT studies, a total of 745 samples, the life-quality scores between the experimental group and the control group were analyzed via meta-analysis. There was obvious heterogeneity of life-quality scores among the included research data (chi^2^ = 104.15, df = 4, *P* < 0.00001, *I*^2^ = 96%). It was indicated that there was obvious heterogeneity among the included research data. According to the results of this analysis, it was considered that there is a statistical difference in the score of quality of life between peritoneal dialysis and hemodialysis in patients with end-stage renal disease, indicating that the score of quality of life of patients with end-stage renal disease treated by peritoneal dialysis is significantly better than that of hemodialysis. All the results are shown in Figure 5.

## 4. Discussion

Chronic kidney disease (CKD) refers to renal structural and functional disorders caused by various causes for more than 3 months, including pathological damage with normal and abnormal glomerular filtration rate, abnormal blood or urine composition, and abnormal imaging examination, or decreased glomerular filtration rate (GFR) for more than 3 months (<60 ml/min) [25]. Due to the aging of the population and the increase in the incidence of chronic diseases such as diabetes, hypertension, and metabolic syndrome, the number of CKD patients is increasing rapidly. The prevalence rate of CKD in adults in mainland China is about 11% [26]. Previous data from the US Renal Data System (USRDS) in 2018 showed that the prevalence rate of adult CKD was about 15% [27]. With the deterioration of renal function, CKD will eventually progress to end-stage renal disease (ESRD). ESRD refers to the end stage of all kinds of CKD or GFR < 15 ml/(min · 1.73 m^2^) [28], requiring renal replacement therapy (RRT) CKD. It is estimated that 3 million people have ESKD, and their lives depend on dialysis treatment [29].

At present, some statistics have suggested that the proportion of patients with end-stage kidney disease receiving HD treatment is significantly higher than that receiving PD treatment. Because hemodialysis patients are operated on by professional nurses, the treatment process is completed in a short period of time [30]. First of all, hemodynamic changes of patients with end-stage renal disease in a short period of time during hemodialysis make patients feel exhausted and the process unbearable [31]. Secondly, activity travel is seriously affected after hemodialysis treatment. A questionnaire survey showed that HD patients would rather shorten their survival rate by 2 years than be restricted in travel [32]. In addition, the most prominent problem of HD patients with end-stage renal disease is the solution of the vascular pathway. A central venous catheter is commonly used at present, and its high incidence of thrombosis and infection is a prominent problem in dialysis patients using this vascular pathway [33]. At the same time, a long-time indwelling central venous catheter may increase the risk of local venous stenosis. Therefore, the use of the central venous catheter in patients is greatly limited. Recent studies have shown that the ideal vascular pathway for hemodialysis patients is still autologous arteriovenous fistula, while in patients with end-stage renal disease, atherosclerosis is obvious, and the proportion of diabetes mellitus and heart failure is significantly increased. At the same time, the mature time of arteriovenous fistula may be longer than its survival time [34], which affects the utilization rate of autologous arteriovenous fistula in some patients with end-stage renal disease.

Peritoneal dialysis is widely used all over the world. Compared with hemodialysis indicators, peritoneal dialysis has a significant effect on the improvement of renal function and quality of life of patients. A recent study found that nephrologists can make 25%-30% of PD patients better manage PD treatment, which is much higher than that observed in clinical practice [35]. At the same time, there are still many obstacles in elderly patients with peritoneal dialysis [36, 37]. It can easily lead to negative emotion and increase the risk of complications. When 61% of elderly patients can choose PD or HD treatment, only 10% of elderly patients choose HD treatment [38, 39]. In Europe, although HD treatment is relatively common, elderly patients choosing HD treatment is still significantly less than PD treatment. Early studies have pointed out that for most ESRD patients who receive renal replacement therapy for the first time. 93%-98% of them choose peritoneal dialysis therapy and only 2%-5% of them choose blood therapy [40]. Similarly, elderly patients have been treated with PD successfully under the policy of “PD first” in Hong Kong. As of March 2007, some 80% ESRD patients were treated with PD with an average age of 62.3 years [41–43]. This is because PD treatment also has some advantages for elderly patients. Some European countries began to implement the strategy of adjuvant PD therapy (including professional nurse-assisted therapy and automated peritoneal dialysis machine therapy), which greatly improved the life quality and survival rate of elderly PD patients [44, 45].

Due to the improvement of survival rate of ESRD patients, life quality and renal function as evaluation indicators of dialysis treatment have become the focus of attention of patients and their families. ESRD patients with a long treatment cycle often have tension, anxiety, or even depression. In addition, for patients who had been on dialysis for more than 3 years, RRF and daily diet decreased and exercise was limited, resulting in a decline in the quality of life of patients. The goal of quality of life is not to eliminate the disease but to adjust the patient's physical condition and change the patient's lifestyle [46–48]. Several studies have found no significant difference in mortality among different dialysis methods which further suggest that the potential benefits of quality of life may directly promote the choice of initial dialysis methods [49–51]. The quality of the renal function index is closely related to the better quality of life and higher survival rate of ESRD patients. Many studies have found that in both HD and PD patients. The survival rate of patients with renal function is higher than that of patients without renal function, and the quality of life of patients with renal function is better than that of patients without renal function. Because of the different dialysis characteristics of HD and PD, some studies have shown that PD can protect patients' renal function better than HD [52, 53]. In PD patients, the loss of renal function can be slowed down by using renin-angiotensin-aldosterone system blockers and diuretics. There are some limitations in this study. First of all, the sample size of the references included in this study is small, and they all belong to single-center research; there is a certain deviation. In the future research, we will carry out a large sample of prospective studies and hopefully draw more valuable conclusions.

## 5. Conclusion

Compared with hemodialysis in the treatment of end-stage renal disease, the renal function and life quality of patients with peritoneal dialysis are better than those of hemodialysis patients. Further studies and follow-up with higher methodological quality and longer intervention time are still needed for further verification.

## Figures and Tables

**Figure 1:** Risk of bias chart.

**Figure 2:** Summary chart of risk bias.

**Figure 3:** Forest plot of meta-analysis of Scr indicator. Note: Chi^2^: chi-square test; df: degree of freedom; P: significant *P* value; I^2^: heterogeneity test.

**Figure 4:** Forest plot of meta-analysis of BUN indicators. Note: Chi^2^: chi-square test; df: degree of freedom; P: significant *P* value; I^2^: heterogeneity test.

**Figure 5:** Forest plot of meta-analysis of quality of life score. Note: Chi^2^: chi-square test; df: degree of freedom; P: significant *P* value; I^2^: heterogeneity test.

**Table 1:** The basic characteristics of literature.

Include the literature	Year of publication	*N* (*C*/*T*)	Intervention method		Outcome index	Experimental time	Whether it is random or not	Whether it is blind or not
			*C*	*T*				
Zhu Xueli	2020	100/100	Hemodialysis	Peritoneal dialysis	③	6 months	Yes	No
Zhang Qingjuan	2012	35/30	Hemodialysis	Peritoneal dialysis	③	6 months	Unknown	No
Dong Jingying	2021	45/41	Hemodialysis	Peritoneal dialysis	① ②	6 months	No	No
Liu Boying	2020	52/52	Hemodialysis	Peritoneal dialysis	① ②	6 months	Yes	No
Li Rui	2020	50/50	Hemodialysis	Peritoneal dialysis	① ② ③	1 year	Yes	Yes
Zheng Yiting	2018	46/46	Hemodialysis	Peritoneal dialysis	① ② ③	1 year	No	No
Duan Qian	2018	55/43	Hemodialysis	Peritoneal dialysis	① ② ③	1 year	No	No

① Serum creatinine; ② BUNTIX; ③ quality-of-life score.

## Data Availability

The datasets used and analyzed during the current study are available from the corresponding author upon reasonable request.
